The article "Effect of Levothyroxine Sodium Tablets on Pregnancy Outcome and Offspring Development Quotient of SCH during Pregnancy" was published in 2022. Journal: J Healthc Eng.

# Effect of Levothyroxine Sodium Tablets on Pregnancy Outcome and Offspring Development Quotient of SCH during Pregnancy

**DOI:** 10.1155/2022/9001881

**Published:** 2022-03-28

**Authors:** Xiaoling Qian, Yunying Sun, Xiaohua Xu

**Affiliations:** Department of Endocrinology, Haining People's Hospital, Haining 314400, Zhejiang, China

## Abstract

**Objective:**

To investigate the effect of levothyroxine sodium tablets (L-T4) on pregnancy outcome and offspring development quotient in patients with subclinical hypothyroidism (SCH) during pregnancy. *Material and Methods.* Pregnant women with gestational age less than 12 weeks who underwent the first prenatal examination in our hospital from January 2019 to December 2019 were prospectively selected as subjects. According to the level of thyroid hormone in pregnant women, they were divided into the treatment group (n = 63) and received L-T4 treatment, untreated group (n = 64), and control group (n = 54). Three groups of pregnancy outcomes, children's physical development, and the development of offspring were compared at when one full year of life.

**Results:**

After treatment, the contrast difference of the three groups about abortion and gestational diabetes mellitus (GDM) was statistically significant (*P* < 0.05). The abortion rate and gestational diabetes mellitus (GDM) in the untreated group were higher than those in the control group (*P* < 0.05). The contrast difference of the treatment group and control group about abortion and gestational diabetes mellitus (GDM) is not statistically significant (*P* > 0.05); The contrast difference of the three groups about a filial generation at birth and one-year-old body length is not statistically significant (*P* > 0.05). The contrast difference between the three groups of individual children who are one-year old having the individual action energy, material ability, speech ability, and human ability is statistically significant (*P* < 0.05). One-year-old developmental quotient (DQ) of the treatment group and control group was higher than that of the untreated group (*P* < 0.05); the Pearson correlation analysis showed that the treatment group TSH levels have no correlation between the offspring developmental quotient (DQ) level of one-year-old children (*P* > 0.05).

**Conclusion:**

Levothyroxine sodium tablets (L-T4) can not only improve the pregnancy outcome of patients with SCH during pregnancy but also play a positive role in improving the neurointellectual development of their offspring.

## 1. Introduction

Subclinical hypothyroidism during pregnancy is an endocrine disease, which is caused by the decrease of thyroid hormone secretion and the increase of thyroid-stimulating hormone. It is mostly diagnosed by laboratory examination. The maternal thyroid is in a special physiological period during pregnancy, and the thyroid level plays a key role in the maintenance of normal pregnancy and fetal growth and development. Early studies have shown that [1, 2] thyroid hormone deficiency during pregnancy is not only related to pregnancy complications and obstetric outcomes such as spontaneous abortion, preterm delivery, and postpartum hemorrhage but also related to neurointellectual development disorders in offspring. Subsequent studies on subclinical hypothyroidism (SCH) during pregnancy and pregnant women and their offspring have attracted wide attention, and several researchers [3, 4] think it is very important to keep the gestational thyroid function in an ideal reference value range. China's guidelines recommend that [5] the replacement and supplementary treatment of levothyroxine sodium tablets (L-T4) is the key measure in the case of thyroid hormone deficiency during pregnancy; the European Thyroid Association (ETA) [6] believes that all pregnant women with SCH during pregnancy should be treated with levothyroxine sodium tablets (L-T4); the American Thyroid Association (ATA) [7] recommends L-T4 treatment for SCH in pregnant women with resistance to thyroid peroxidase antibodies (TPO-Abs) positive. Patients with thyroid peroxidase antibodies (TPO-Abs) negative neither recommend nor oppose treatment, which will undoubtedly affect the judgment of SCH treatment during pregnancy.

The article "Effect of Levothyroxine Sodium Tablets on Pregnancy Outcome and Offspring Development Quotient of SCH during Pregnancy" was published in 2022. Journal: J Healthc Eng.

The current study shows that levothyroxine sodium tablets are the first choice for the treatment of subclinical hypothyroidism during pregnancy and can replace thyroid hormone [8]. Evidence-based clinical evaluation studies have shown that levothyroxine replacement therapy can reduce the risk of adverse pregnancy outcomes in women with subclinical hypothyroidism (SCH) [9]. However, the current views on the treatment of subclinical hypothyroidism during pregnancy with levothyroxine sodium tablets are not completely consistent. Therefore, it is particularly important to take effective measures to maintain thyroid function during pregnancy in the ideal reference value range [10, 11]. In order to further clarify whether L-T4 treatment can benefit pregnant patients with SCH, this study analyzed the pregnancy outcome, offspring physique, and development quotient, in order to explore whether L-T4 intervention can play a role in eugenics and fertility, and provide a new theoretical basis for the treatment of pregnant patients with SCH.

## 2. Material and Statistical Analysis

### 2.1. General Information

Prospective pregnant women whose gestational weeks were less than twelve weeks were prospectively selected from January 2019 to December 2019 for the first antenatal examination. The inclusion criteria are as follows: (i) it meets the diagnostic criteria of the Guidelines for Diagnosis and Treatment of Thyroid Diseases in Pregnancy and Postpartum [12]; (ii) normal singleton pregnancy; and (iii) no previous history of adverse pregnancy. The exclusion criteria are as follows: (i) merging other serious diseases affecting the endocrine system; (ii) merging family history of thyroid disease; and (iii) assisted reproductive technology. This information was reviewed by the Hospital Ethics Committee; pregnant women and their families signed informed consent, and they were qualified for long-term followup. According to the level of thyroid hormones during pregnancy, patients were divided into the treatment group (*n* = 63) [2.5 mIU/L < Thyroid Stimulating Hormone (TSH) ≦ 4.0 mIU/L, with TPO-Ab positive reaction; TSH ＞ 4.0 mIU/L], untreated group(*n* = 64) (2.5 mIU/L < TSH ≦ 4.0 mIU/L, with TPO-Ab negative reaction), and control group (*n* = 54) (TSH ≦ 2.5 mIU/L). Among the three groups, there was no statistically significant difference when compared in terms of baseline data (*P* > 0.05) (Table 1).

The article "Effect of Levothyroxine Sodium Tablets on Pregnancy Outcome and Offspring Development Quotient of SCH during Pregnancy" was published in 2022. Journal: J Healthc Eng.

### 2.2. Method

#### 2.2.1. Untreated Group and Control Group

Regular visits were conducted according to the requirements of pregnancy health care, and pregnancy complications and obstetrical outcomes were observed.

#### 2.2.2. Treatment Group

After confirming the diagnosis of SCH, L-T4 (China Associate Pharmaceutical Co., LTD; H20010008; 25 ug) was given immediately according to the thyroid function, and the initial oral dose was determined according to the elevated degree of TSH; according to the Guidelines for Diagnosis and Treatment of Thyroid Diseases in Pregnancy and Postpartum (2nd edition), it is recommended that TSH > The upper limit of pregnancy-specific reference value is 2.5 mIU/L, initial dose 50 *μ*g/d; TSH > 8.0 mIU/L, initial dose 75 *μ*g/d; once a day, the tablet was taken in an empty stomach in the morning. During this period, the dose was adjusted according to the treatment target of serum TSH. Early, middle, and late pregnancy TSH levels were maintained at 0.1∼2.5 mIU/L, 0.2∼3.0 mlU/L, and 0.3∼3.0 mIU/L. The medication was stopped at the end of pregnancy, and the thyroid function was reexamined regularly to return to the normal range. The medication is stopped at the end of pregnancy, thyroid function is regularly rechecked to return to the normal range, and pregnancy complications, obstetric outcomes, and the neurointellectual development of offspring are followed up at the age of one year through outpatient service, telephone, and WeChat.

The article "Effect of Levothyroxine Sodium Tablets on Pregnancy Outcome and Offspring Development Quotient of SCH during Pregnancy" was published in 2022. Journal: J Healthc Eng.

### 2.3. Observation Index

#### 2.3.1. Pregnancy Outcomes

Abortion, gestational diabetes mellitus (GDM), gestational hypertension, preterm birth, and full-term small kind were observed.

#### 2.3.2. Children Physique Level

The heel blood of the offspring was collected three days after birth; the TSH level was measured by an automatic biochemical immune analyzer (model: Hitachi 70802), and the basic data such as the body length and weight of the offspring at birth and one-year old were collected.

#### 2.3.3. Level of Offspring Development Quotient

Using Gesell development scale [13], a specially assigned person was assigned to evaluate the neurointelligence development of the offspring at the age of 1 year, and the abilities of individual action ability, material ability, speech ability, and human ability were evaluated for 30 minutes. Development quotient = Developmental age/Actual age × 100.

### 2.4. Quality Control

The inclusion criteria and exclusion criteria were strictly implemented, the research protocol is reviewed and revised, and relevant personnel was needed to be participated in training to ensure the accuracy and integrity of clinical data, and the parallel double-entry method is used for statistical data.

### 2.5. Statistical Processing

Epidate software and spss20.0 software were used to analyze the data, the measurement data in line with normal distribution were expressed in ($\bar{\chi }\pm s$), `_`_repeated ANOVA was used for multi group comparison, and independent sample *t* test was used for pairwise comparison. The counting data were expressed in the form of number of cases/composition ratio *n*(%), use of *χ*^2^ inspection, pairwise comparison, correction by Bonferroni method, and setting the correction level as 0.017 (0.05/3). The rank sum test was used for rank data; Pearson correlation analysis was used to analyze the correlation between the TSH level of pregnant women in the treatment group and one-year-old development quotient level of their offspring. *P* < 0.05 indicates that the difference is significant.

## 3. Results

### 3.1. Comparison of Pregnancy Outcomes among Three Groups of Pregnant Women

The difference between the three groups of abortion and gestational diabetes mellitus was statistically significant (*P* < 0.05); the abortion rate and gestational diabetes mellitus (GDM) in the untreated group were higher than those in the control group (*P* < 0.05). The difference between the treatment group and the control group in the abortion rate and gestational diabetes mellitus was not statistically significant (*P* > 0.05). The difference between the three groups in preterm birth, full-term small sample, and gestational hypertension was not statistically significant (*P* > 0.05) (Table 2).

The article "Effect of Levothyroxine Sodium Tablets on Pregnancy Outcome and Offspring Development Quotient of SCH during Pregnancy" was published in 2022. Journal: J Healthc Eng.

### 3.2. Three Groups of Children Physical Development Index Contrast

There was no statistically significant difference weight contrast (*P* > 0.05) in three groups of children who were born and one full year of life long (Table 3).

### 3.3. Comparison of One-Year-Old Development Quotient of Three Groups of Offspring

The difference between individual action energy, material ability, speech ability, and human ability among the three groups was not statistically significant (*P* < 0.05). The development quotient at the age of one in the treatment group and the control group was higher than that in the untreated group (*P* < 0.05) (Table 4).

### 3.4. The Correlation between TSH Level of Pregnant Women in the Treatment Group and One-Year-Old Development Quotient Level of Their Offspring

According to Pearson correlation analysis, the difference between the TSH level of pregnant women in the treatment group and one-year-old development quotient level of their offspring had no correlation (*P* > 0.05) (Table 5).

## 4. Discussions

Thyroid hormone is a key regulator of metabolism. In order to meet the needs of the tissue, the production of thyroid hormone is regulated by the hypothalamic-pituitary-thyroid (HPT) axis. During the intrauterine development of the HPT axis, the fetal thyroid is not yet mature and mainly depends on placental metastasis to maintain the thyroid function [14]. Basic research confirmed [15, 16] the important role of maternal thyroid hormone in the first half of fetal brain development, which aroused strong interest in the relationship between maternal thyroid hormone and fetal brain development in many disciplines. Recent studies show [17] the thyroid hormone lack of brain development and brain patterns to the influence of different levels, especially brain morphology, and it has been confirmed that the relative gray matter volume and cortex thickness of the brain are positively correlated with the development quotient, which makes the early screening and treatment of SCH during pregnancy pay more attention. L-T4 replacement therapy is the preferred drug for SCH during pregnancy at present. TSH level can be controlled within a reasonable range according to the target value, which makes L-T4 therapy gradually pay attention in patients with gestational SCH.

Current studies believe that [18] SCH during pregnancy can increase adverse pregnancy outcomes such as preterm delivery, abortion, and pregnancy complications [19]. A randomized controlled trial [20] reduced adverse pregnancy outcomes after L-T4 treatment for women with TSH >2.5 mIU/L and TPO-Ab positive pregnancy for nine weeks. Then, a MATE analysis showed that [21] L-T4 treatment can reduce 50% risk for spontaneous abortion patients with SCH. This study also shows that the abortion rate and gestational diabetes mellitus in the untreated group were higher than those in the control group, but in Kianpour and other studies [22], the rate of spontaneous abortion in the SCH group during pregnancy was lower than that in the untreated group after receiving L-T4 treatment, but the difference was not statistically significant. Levothyroxine, vitamin B12, and folic acid can be used to treat pregnant women with SCH. In addition, regular monitoring of blood glucose level, blood lipid and homocysteine level, and intervention of weight gain during pregnancy can reduce the adverse effect of SCH on the pregnancy outcome [23]. We believe that the reason for the inconsistent pregnancy outcome after L-T4 treatment is that there are differences in genetic background and living environment among different research populations, and the limited range of normal reference value of TSH in research diagnosis is inconsistent. Nevertheless, overall, L-T4 may be beneficial in reducing these complications in patients with SCH pregnancy.

The article "Effect of Levothyroxine Sodium Tablets on Pregnancy Outcome and Offspring Development Quotient of SCH during Pregnancy" was published in 2022. Journal: J Healthc Eng.

The early and middle trimester of pregnancy is the first rapid stage of fetal neural development, which mainly supplies fetal thyroid hormone through placental transport [24]. If the level of thyroid hormone is deficient at this stage, it will lead to the maturation disorder of fetal cortical pyramid cells and glial cells. The involvement of thyroid hormone in the occurrence and formation of neurons in the hippocampus and somatosensory area cortex has been confirmed in previous studies [25]. A follow-up survey of the offspring of pregnant women with subacute hypothyroidism at 20 weeks of pregnancy found that [26], compared with the 30-month exercise and intelligence scores of the offspring of normal pregnant women, the exercise and intelligence scores of the offspring of pregnant women with subacute hypothyroidism were significantly lower. Maternal TPO Ab titer and TSH level were risk factors affecting offspring's motor and intelligence scores. Subsequently, in order to further explore whether gestational SCH will have a long-term impact on the neurointelligence development of their offspring, some scholars found that [27] SCH during pregnancy will have an impact on the intelligence development of their offspring at the age of seven and eight, and compared with pregnant women with normal thyroid function, the intelligence quotient (IQ) of the offspring of untreated SCH pregnant women is reduced by seven percentage points, and the exercise ability is also affected to a certain extent; this supports this conclusion.

The article "Effect of Levothyroxine Sodium Tablets on Pregnancy Outcome and Offspring Development Quotient of SCH during Pregnancy" was published in 2022. Journal: J Healthc Eng.

The intellectual development of offspring of subclinical hypothyroidism with TPOAb-negative during pregnancy is associated with TSH level. Standardized treatment of subclinical hypothyroidism with TPOAb-negative during pregnancy and control of TSH level at 4.0∼10.0 mIU/L before 8 weeks of pregnant women can significantly improve the intellectual development level of offspring at 2 years old [28]. The results of this study show that the one-year-old development quotient (DQ) of the treatment group and the control group is higher than that of the untreated group, indicating that L-T4 treatment is of positive significance. L-T4 treatment during pregnancy can avoid the neurointelligence damage of offspring caused by maternal thyroid hormone deficiency to a certain extent. Thyroid hormone affects the function and structure of the brain. In a study of hypothyroidism during pregnancy in rats [29], it can interfere with the spatial learning and memory function of young rats. It is also found that some protein levels in hippocampus have changed, and the above damage can be reversed by early L-T4 treatment and functional exercise. In addition, this study uses Pearson correlation analysis to show that there was no correlation between TSH level during pregnancy and the one-year-old development quotient level of offspring in the treatment group (*P* > 0.05), which further explained that L-T4 intervention for pregnant women with hypothyroidism during pregnancy may play a positive role in improving the development of neurointelligence of their offspring at one-year old. It is possible that after the intervention of L-T4, the thyroid function of pregnant women is maintained within the control target during pregnancy, which makes up for the deficiency of thyroid hormone during pregnancy, ensures the differentiation and development of nervous system in the fetal stage, and does not cause damage to the neurointelligence of the offspring at the age of one.

## 5. Conclusion

In conclusion, levothyroxine sodium tablets (L-T4) can not only improve the pregnancy outcome of pregnant SCH patients but also play a positive role in improving the development of neurointelligence of their offspring. Therefore, early screening of maternal thyroid function and reasonable treatment will be helpful for pregnant women and their offspring. This study also has some shortcomings. Firstly, the sample size is relatively small, which may lead to bias in the research results; there are deficiencies in the setting and complexity of relevant data sample sets. Secondly, only the developmental quotient level of the offspring at the age of 1 year is explored. The effect of levothyroxine sodium tablets on the long-term developmental quotient of the offspring still needs to be verified by large-scale and prospective studies to optimize the treatment scheme.

The article "Effect of Levothyroxine Sodium Tablets on Pregnancy Outcome and Offspring Development Quotient of SCH during Pregnancy" was published in 2022. Journal: J Healthc Eng.

## Figures and Tables

**Table 1:** Three groups of baseline data comparison [*n*, ($\bar{\chi }\pm s$)].

Baseline data	Treatment group (*n* = 63)	Untreated group (*n* = 64)	Control group (*n* = 54)	*χ* ^2^/*F* value	*P* value
Age (years old)	28.39 ± 3.98	29.01 ± 3.04	28.56 ± 3.46	0.525	0.592
Both the gestational age (week)	14.23 ± 2.36	13.96 ± 2.87	14.42 ± 2.64	0.458	0.634
Pregnancy body mass index (kg/m^2^)	22.63 ± 1.63	22.49 ± 1.74	22.58 ± 1.69	0.112	0.894
Home place (*n*, %)					
City	30 (47.62)	34 (53.13)	34 (62.96)	2.799	0.247
Rural	33 (52.38)	30 (46.87)	20 (37.04)		
Number of years of education (years)	10.25 ± 2.65	10.27 ± 2.51	10.30 ± 2.14	0.006	0.994

**Table 2:** Comparison of pregnancy outcomes among three groups of pregnant women (*n*, %).

Group	Case number	Abortion	Premature delivery	Full-term small sample	Gestational hypertension	Gestational diabetes mellitus (GDM)
Treatment group	63	3 (4.76)	3 (4.76)	4 (6.35)	4 (6.35)	4 (6.35)
Untreated group	64	7 (10.94)	6 (9.34)	5 (7.81)	6 (9.34)	9 (14.06)
Control group	54	0 (0.00)	1 (1.85)	1 (1.85)	1 (1.85)	1 (1.85)
*χ* ^2^ values		6.820	3.284	2.119	2.917	6.379
*P* values		0.033	0.194	0.347	0.233	0.041

**Table 3:** Comparison of physical development indexes of three groups of offspring ($\bar{\chi }\pm s$).

Group	Case number	Body length (cm)		Weight (kg)	
		In birth	1-year old	In birth	1-year old
Treatment group	60	49.32 ± 2.01	74.63 ± 2.96	3.26 ± 0.24	8.26 ± 1.69
Untreated group	57	49.01 ± 1.93	73.69 ± 2.87	3.22 ± 0.28	8.11 ± 1.72
Control group	54	49.39 ± 2.03	75.01 ± 2.89	3.33 ± 0.27	8.32 ± 1.83
*F* values		0.583	2.377	2.470	0.215
*P* values		0.560	0.096	0.088	0.806

**Table 4:** Comparison of 1-year-old development quotient of three groups of offspring ($\bar{\chi }\pm s$, minute).

Group	Case number	Individual action energy	Material ability	Speech ability	Human ability
Treatment group	60	102.32 ± 12.24	101.25 ± 12.01	90.23 ± 10.25	102.35 ± 12.34
Untreated group	57	96.67 ± 10.45	96.35 ± 10.05	86.35 ± 9.37	96.34 ± 11.88
Control group	54	104.27 ± 11.23	102.58 ± 12.22	92.78 ± 10.24	104.24 ± 12.02
*F* values		6.794	4.612	5.887	6.548
*P* values		0.001	0.011	0.003	0.002

**Table 5:** The correlation between TSH level of pregnant women in the treatment group and 1-year-old development quotient level of their offspring.

Development quotient	TSH level of pregnant women	
	*r*	*p*
Individual action energy	−0.165	0.209
Material ability	0.018	0.890
Speech ability	−0.033	0.805
Human ability	−0.240	0.065

The article "Effect of Levothyroxine Sodium Tablets on Pregnancy Outcome and Offspring Development Quotient of SCH during Pregnancy" was published in 2022. Journal: J Healthc Eng.

## Data Availability

All data related to this study can be obtained from the corresponding author. This study is fully consistent with journal data availability.
